The article "From fever to immunity: A new role for IGFBP‐6?" was published in 2018. Journal: J Cell Mol Med.

# From fever to immunity: A new role for IGFBP‐6?

**DOI:** 10.1111/jcmm.13738

**Published:** 2018-08-17

**Authors:** Arcangelo Liso, Nazzareno Capitanio, Roberto Gerli, Massimo Conese

**Affiliations:** ^1^ Department of Medical and Surgical Sciences University of Foggia Foggia Italy; ^2^ Department of Clinical and Experimental Medicine University of Foggia Foggia Italy; ^3^ Department of Medicine University of Perugia Perugia Italy

**Keywords:** cancer microenvironment, dendritic cells, fever, immune system, inflammation, mitochondrial metabolism, neutrophils, T cells

## Abstract

Fever is a fundamental response to infection and a hallmark of inflammatory disease, which has been conserved and shaped through millions of years of natural selection. Although fever is able to stimulate both innate and adaptive immune responses, the very nature of all the molecular thermosensors, the timing and the detailed mechanisms translating a physical trigger into a fundamental biological response are incompletely understood. Here we discuss the consequence of hyperthermic stress in dendritic cells (DCs), and how the sole physical input is sensed as an alert stimulus triggering a complex transition in a very narrow temporal window. Importantly, we review recent findings demonstrating the significant and specific changes discovered in gene expression and in the metabolic phenotype associated with hyperthermia in DCs. Furthermore, we discuss the results that support a model based on a thermally induced autocrine signalling, which rewires and sets a metabolism checkpoint linked to immune activation of dendritic cells. Importantly, in this context, we highlight the novel regulatory functions discovered for IGFBP‐6 protein: induction of chemotaxis; capacity to increase oxidative burst and degranulation of neutrophils, ability to induce metabolic changes in DCs. Finally, we discuss the role of IGFBP‐6 in autoimmune disease and how novel mechanistic insights could lead to exploit thermal stress‐related mechanisms in the context of cancer therapy.

## 1 INTRODUCTION

The immune system of vertebrates is organized to respond either to pathogens or to *noxae* that cause damage or trauma. In both cases, the organism needs to activate a complex system composed of warning signals, cellular receptors to respond, signalling pathways and outputs in the form of physiological responses. Endogenous signals that alert the immune system on cell and tissue damage are called “alarmins,” whereas pathogen‐associated molecular patterns (PAMPs) flag the presence of intruding pathogens. Together, alarmins and PAMPs constitute the larger family of damage‐associated molecular patterns, or DAMPs.^1^

The article "From fever to immunity: A new role for IGFBP‐6?" was published in 2018. Journal: J Cell Mol Med.

It is well‐known that exogenous PAMPs are recognized by cells of the innate and adaptive immune systems through quite a number of receptors, called pattern recognition receptors (PRRs), which include Toll‐like receptors, RIG‐I‐like receptors, NOD‐like receptors and C‐type lectin receptors.^2^ On the other hand, alarmins are either rapidly released upon cells undergoing necrosis or are secreted by immune cells. As for PAMPs, they recruit and activate cells of the immune system, as PAMPs are recognized by cellular receptors, especially expressed by DCs, and finally should induce repair of the tissue that was damaged by direct insult or secondary inflammation. The prototypical alarmin molecule is represented by high mobility group box 1 (HMGB1), comprising heat shock proteins (HSPs) and cytokines such as IL‐1α, IL‐33, IL‐16.^1^, ^3^, ^4^, ^5^, ^6^, ^7^

The insulin‐like growth factor (IGF) system is essential for growth and development, and it has been implicated in several diseases.^8^ IGF activity is precisely regulated by a family of six high‐affinity IGF binding proteins (IGFBPs).^9^ Moreover, IGFBPs bind non‐IGF ligands in the extracellular space, cell membrane, cytoplasm and nucleus, thereby modulating cell proliferation, survival and migration in an IGF‐independent manner.^10^

Fever, a hallmark of infection and inflammation, is comprised of physiological and neurological circuitries that have been conserved in warm and cold‐blooded vertebrates for over 600 million years of evolution. Significantly, fever represents a fundamental systemic response which stems from the recognition of PAMPs by PRRs, determining the production of cytokines, among which IL‐6 is the most important mediator for fever induction and orchestrating lymphocyte trafficking to lymphoid organs.

In this review, we have highlighted new findings related to the effect of fever‐range hyperthermia on the immune system, in particular DC activation and metabolic reprogramming, monocyte and T cell chemotaxis, and neutrophil activation. A novel role for insulin‐like growth factor binding protein 6 (IGFBP‐6) is also discussed in this hyperthermia‐induced rewiring of the immune system. Implications for the inflammatory response in autoimmune diseases and cancer are also presented.

## 2 HYPERTHERMIA INDUCES SPECIFIC GENETIC AND METABOLIC REPROGRAMMING OF DENDRITIC CELLS

Febrile temperatures (ie, ranging from 38‐41°C; ΔT~1‐4°C above baseline) boost the effectiveness of the immune response during infections by stimulating both the innate and adaptive arms of the immune system.^11^ Indeed, hyperthermia elicits neutrophil functions, DC maturation and DC ability to stimulate T cells, enhance T cell trafficking through lymph nodes and effector T cell differentiation. AS fever is known to confer a survival advantage by warding off attack by invading pathogens, it is crucial to understand in greater details how it activates sensors, transducing pathways and effector mechanisms.

The article "From fever to immunity: A new role for IGFBP‐6?" was published in 2018. Journal: J Cell Mol Med.

A wealth of data on the role of metabolic pathways controlling immune cell function have shed new light on both the innate and adaptive immune response, and led to the discovery of “immunometabolism” as an important area of research.^12^, ^13^, ^14^ Notably, metabolic processes (eg, glycolysis, the Krebs cycle and fatty acid metabolism) have all been shown to have highly specific effects on DCs function^15^, ^16^ and, most importantly, alterations of either one of these metabolic pathways have been shown to dramatically alter the functioning of these cells in ways not simply linked to energy production or general biosynthesis.^17^

Recently, we explored how a short‐term mild hyperthermal activation of monocyte‐derived dendritic cells (MoDCs) intertwined with changes in the metabolic phenotype.^18^ In this context, we focused mainly on the mitochondrial respiratory and oxidative phosphorylation (OxPhos) activity given their pivotal role in the cell bioenergetics. In summary, we found that: (i) fever‐like hyperthermia (3 hours exposure at 39°C) induces cytokine release in MoDCs, (ii) hyperthermia rewires MoDC metabolism by inhibiting mitochondrial OxPhos, (iii) the process is linked to interplaying nitric oxide (NO) and reactive oxygen species (ROS) release and mitochondrial (mt) Ca2+ accumulation, (iv) antioxidants or mitochondrial Ca^2+^ uniporter (MCU) inhibition prevents mt‐OxPhos inhibition and cytokine release. Figure 1 depicts the main findings of this study.

**Figure 1:** Effect of mild hyperthermic stress on dendritic cells. The picture shows schematically the main results of a study^18^ carried out on cultured human monocyte‐derived dendritic cells (MoDCs) exposed for 3 h from 37 to 39°C. The major outcomes, observed in hyper‐thermic MoDC appear to involve the mitochondrial oxidative metabolism and consisted in decreased activity of the mitochondrial respiratory chain and consequent oxidative phosphorylation (OxPhos), enhanced production of reactive nitrogen and oxygen species (RONS) and overload of intramitochondrial (mt) Ca^2+^ ions. This was accompanied with increased glycolysis, suggesting metabolic rewiring, and release of pro‐inflammatory cytokines. All the above reported effects were re‐capitulated in normothermic MoDCs exposed to the conditioned medium of the 39°C‐treated cells thus suggesting the involvement of secretome‐contained factors. On the basis of results of a transcriptome study performed on the same cells under identical hyperthermic conditioning,^21^ HSP70 and IGFBP‐6 are indicated as putative candidates acting via an autocrine mechanism. The shown protein structures of IGFBP‐6 and HSP70 were taken from the RCSB‐protein data bank (http://www.rcsb.org/)

Strikingly, the same hyperthermic conditioning, that in MoDCs cause a significant change in the mitochondrial physiology, resulted in no change at all in mitochondrial respiratory activity of undifferentiated monocytes, which mainly rely on glycolysis.^19^

The article "From fever to immunity: A new role for IGFBP‐6?" was published in 2018. Journal: J Cell Mol Med.

And in fact, in monocytes we observed no variation in OxPhos‐related respiratory activity and of the redox and Ca^2+^ homoeostasis. This clearly points to a cell‐specific sensitivity of the mitochondrial activity to the thermal stress and suggests that metabolic pathways under thermal control are of pivotal importance in DCs physiology. Our priority in fact has been to study DCs‐specific response to hyperthermia as a mean to better understand fundamental mechanisms controlling immunity.

Importantly, re‐conditioning of the 39°C‐treated MoDCs to normothermia did not appreciably recover the mitochondria‐related activities showing the irreversible nature of this observation. Again this fact suggests that response to fever in DCs is a fundamental and solid process which rapidly activates complex and important pathways in DCs, not easily inhibited after activation.

As activation of immune‐competent cells is also known to be accompanied with changes in the cell secretome,^20^ we tested if release of factors by thermally stressed MoDCs might contribute to the observed alterations of the metabolic phenotype. Insightfully, incubation of normothermic MoDCs with the conditioned medium of the 39°C‐treated cells caused a depression of the mitochondrial respiratory activity as well as of the ROS/reactive nitrogen species (RNS) and Ca^2+^ homoeostasis comparable with that attained in thermally challenged MoDCs. The relevance of our findings was even magnified as we discovered that a relatively small number of genes vary in expression upon brief exposure to mild hyperthermia in DCs when we studied a small group of *bona fide* normal subjects. In our hands, IGFBP‐6 was in fact the only specifically up‐regulated under hyperthermic conditions by MoDCs.^21^

Therefore, we explored in our recent publications^21^, ^22^, ^23^ whether recombinant IGFBP‐6 could be part of a comprehensive working model, amenable to experimental validation, of the possible mechanism driving the physical thermal input into a physiological adaptation in MoDCs.

## 3 IGFS AND IGFBP‐6 HAVE MULTIPLE IMPORTANT FUNCTIONS

Insulin‐like growth factors (IGFs) have a key role in normal growth and development,^8^ whereas their deregulation is associated with many diseases, including cancer, diabetes, atherosclerosis and neurodegeneration.^24^ IGF‐I mediates many, but not all, of the growth factor actions, while both IGF‐I and IGF‐II stimulate proliferation, survival and migration of several cell types. IGFs actions are mediated by binding to various receptors, namely IGF type I (IGF‐IR), IGF type II receptor (IGF‐IIR), insulin receptor type A (IR‐A), insulin receptor type B (IR‐B) and hybrid insulin/IGF‐I receptor.^25^ The cation‐independent mannose 6‐phosphate/insulin‐like growth factor receptor (CI‐MPR) is in fact the IGF‐IIR and it is involved in binding of the serine proteinase granzyme B and crucial for the rapid induction of target cell apoptosis by cytotoxic T cells.^26^ Most IGF actions are mediated by the IGF‐IR. This receptor binds IGFs and insulin with the following hierarchical affinity: IG‐I > IGF‐II > insulin.^27^

The article "From fever to immunity: A new role for IGFBP‐6?" was published in 2018. Journal: J Cell Mol Med.

Insulin‐like growth factor actions are regulated by a family of six high affinity binding proteins (IGFBP 1‐6). All IGFBPs have been shown to inhibit the IGF‐associated actions by preventing IGF‐I receptor binding; however, IGF‐independent cellular effects of IGFBPs have also been demonstrated. Strikingly, IGFBP‐6, which is the focus of the present review, binds and inhibit IGFs, with a relatively higher propensity towards IGF‐II than IGF‐I. As for the cognate IGFBP 1‐5, IGFBP‐6 presents two domains at the N‐ and C‐terminal of the 240 amino acids long chain.^25^ The N‐terminal domain is responsible for binding to IGFs, and it is constituted by two subdomains with the one proximal to the N‐terminal showing unstructured features and a set of disulphide bridges not shared with the other IGFBPs. This subdomain is responsible for the higher affinity to IGF‐II. The C‐terminal domain contributes to IGF binding as well as to IGF‐independent actions. The N‐ and C‐domains are connected by a linker domain which is site of post‐translational modifications (Figure 2). IGFBP‐6 is the only IGFBP that preferentially binds IGF‐II over IGF‐I by more than two orders of magnitude.^28^, ^29^, ^30^ IGF‐II exerts its actions through the IGF‐IR, IGF‐IIR and IR‐A.^31^ IGF‐IR mediates many of the biological effects of IGF‐II and shares structural similarities and properties with the insulin receptor. IGF‐IIR/CI‐MPR exhibits the highest affinity for IGF‐II, consists of a single chain, has no tyrosine kinase activity and is involved in internalization and degradation of IGF‐II,^32^ thus acting as a scavenger receptor to regulate extracellular IGF‐II levels. IGF‐II concentration in plasma is 10‐ to 100‐fold higher than that required for its effect in vitro, a consequence of association with the IGFBPs. Notwithstanding its high circulating levels in adult life, IGF‐II is probably more important in regulating embryonic/foetal growth. *IGF2* is an imprinted gene, meaning that one of the two parental alleles of a locus is expressed. Loss of imprinting of *IGF2*, resulting in abnormal expression of IGF‐II, occurs in a number of cancers, sporadic Wilms’ tumour and often in patients with Beckwith–Wiedemann syndrome, characterized in the neonate by overgrowth with risk of developing Wilms’ kidney tumours.^31^ Moreover, IGF‐II is involved in cardiovascular disease, likely because it has been shown to influence the size of atherosclerotic lesions.^33^

The article "From fever to immunity: A new role for IGFBP‐6?" was published in 2018. Journal: J Cell Mol Med.

Here we briefly review the main IGFBP‐6 categories of actions: IGF‐I and IGF‐II dependent, as well as IGF independent functions.

### 3.1 IGF‐I‐dependent actions of IGFBP‐6

Growth hormone (GH) is the major factor stimulating IGF‐I biosynthesis and release, and IGF‐I mediates many, but not all, of its activities.^25^, ^34^ The post‐natal growth of bone and muscles depends on pre‐ and post‐pubertal levels of IGF‐I.^35^ IGFBP‐3 appears to be the main IGFBP regulating the availability of IGF‐I systematically, as most of the IGF‐I and IGF‐II molecules in serum are found in a 150‐kDa ternary complex formed by an IGF, IGFBP‐3 and a glycoprotein known as the acid labile subunit (ALS), all synthesized by the liver.^36^ Not only IGF‐I has endocrine activities, but also autocrine/paracrine ones involved in local growth and response to inflammation.^37^ Human IGFBP‐6 is found predominantly in cerebrospinal fluid (CSF) and serum^38^; however, its physiological significance in regard of IGF‐I at systemic and local levels remains to be elucidated.^39^ Indeed, most studies have failed to show IGF‐I inhibition by IGFBP‐6.^25^

### 3.2 IGF‐II‐dependent actions of IGFBP‐6

IGF‐II has been implicated in mitosis, growth and organ development by paracrine and endocrine pathways in cell culture studies and animal models.^9^, ^37^ The main function of IGFBP‐6 is inhibiting IGF‐II mediated actions concerning cell proliferation, differentiation, migration and survival in many cell lines.^40^, ^41^ In consequence of its inhibitory effect on IGF‐II, IGFBP‐6 has been shown to inhibit the growth and survival of numerous adult and pediatric tumors.

### 3.3 IGF‐independent actions of IGFBP‐6

IGFBP‐6 is capable, however, of actions independent of IGF‐II, including regulation of proliferation, apoptosis, angiogenesis and cell migration.^10^, ^42^ For example, IGFBP‐6 was shown to be effective at attenuating the IGF‐II‐mediated increase in cell contractility of fibroblasts obtained from Dupuytren's disease (DD) patients, while it inhibited DD fibroblast proliferation through mechanisms that are independent of IGF‐II sequestration.^43^

The article "From fever to immunity: A new role for IGFBP‐6?" was published in 2018. Journal: J Cell Mol Med.

### 3.4 Nuclear actions of IGFBP‐6

Some IGFBPs are also nuclear proteins with independent functions from IGFs, and their actions drive the cell fate. IGFBP‐3 and IGFBP‐5 are translocated into the nucleus via the importin‐5 subunit.^44^, ^45^ Both IGFBP‐3 and IGFBP‐5 modulate osteoblast differentiation via interaction with vitamin D receptor (VDR).^46^, ^47^ IGBP‐6 is shuttled to the nucleus via the interaction of its C‐terminal domain with α‐importin, determining apoptosis in rhabdomyosarcoma cells.^48^ Once in the nucleus, IGFBP‐6 regulates osteoblast differentiation by binding to VDR and possibly inhibiting retinoid X receptor (RXR)/VDR heterodimerization.^49^ This interaction brings to the inhibition of VDR‐induced osteocalcin promoter activity and alkaline phosphatase activity (a marker of osteoblast differentiation). Another interaction with nuclear receptors has been highlighted for the thyroid hormone receptor‐α1 (TRα1). Overexpression of IGFBP‐6 suppressed osteoblastic differentiation regulated by TRα1 in the presence of 3,3′,5‐Triiodo‐L‐thyronine.^50^ IGFBP‐6 was demonstrated to bind to the promoter of EGR‐1 (early growth response‐1), a zinc‐finger protein regulator of transcription and thus modulator of cell differentiation and mitogenesis. Overexpression of IGFBP‐6 significantly suppressed the proliferation, invasion and metastatic activity of nasopharyngeal carcinoma cells and increased their apoptosis,^51^ indicating that IGFBP‐6 as a putative tumour suppressor gene. Finally, IGFBP‐6 binds Ku80, that is part of Ku complex involved in the non‐homologous end joining repair, in the cytosol, whereas binds to histone H2Br, which maintains the structural integrity of DNA, in the nucleus.^52^ Overall, these interactions could be part of a mechanism by which IGFBP‐6 regulates apoptosis. Moreover, it could be implicated in other anti‐tumoural effects of IGFBP‐6, such as senescence.^53^, ^54^

The specific impact of IGFBP‐6 on cell metabolism largely relies on its ability to modulate the bioavailability of IGFs thereby antagonizing their receptor(s)‐mediated signalling. A part from their effects on growth and development, IGFs also have insulin‐like effects on metabolism with different tissue‐specific outcomes. However, although IGFs exert an established control on glucose and lipid homeostasis as well as a net anabolic effect on protein metabolism, the molecular mechanisms of their actions are not completely understood. Recent evidences suggest the involvement of the IGF‐IR‐mediated signalling in preserving the mitochondrial structure and function achieved by controlling mitochondrial biogenesis and mitophagy as well as reactive oxygen species homeostasis.^55^, ^56^ In addition to IGFs‐related effects, IGFBPs proved to activate directly receptor‐mediated signaling pathways (see ahead). If and how such direct effects of IGFBPs impact on cell metabolism remains to be established. Intriguingly, one of the recognized IGFBP‐6 receptor is prohibitin‐2 (PBH2).^57^, ^58^ Although PBH2 is located as a single transmembrane helix spanning protein in the cell membrane, the majority of PBH2 is located in a ring‐shaped oligomer in the inner mitochondrial membrane where it functions as a crucial mitophagy receptor.^57^ To notice, intracellular binding partners for IGFBP‐6 have been identified supporting alternative modalities of action thereof.^10^ However, the possible interplay between IGFBP‐6 and the mitochondrial PBH2 has not yet been investigated. Intracellular and intranuclear actions of IGFBP‐6 are depicted in Figure 3.

The article "From fever to immunity: A new role for IGFBP‐6?" was published in 2018. Journal: J Cell Mol Med.

Moreover, more recently other functions of IGFBP‐6 related to the immune system have been discovered (Figure 2), as we found that IGFBP‐6 in vitro acts as a chemoattractant towards neutrophils, monocytes and T cells, but clearly not B cells.^21^, ^23^

**Figure 2:** Extracellular actions of IGFBP‐6. IGFBP‐6 presents both IGF‐dependent and IGF‐independent actions. A subdomain of N‐terminus and the C‐terminal domain likely contribute cooperatively to the IGF‐II‐binding preference.^25^ By binding to IGF‐II and displacing it from its receptors (IGF‐IR, IGF type I receptor; IR‐A, insulin receptor type A; IR/IGF‐IR HR, insulin receptor/IGF receptor hybrid receptor), IGFBP‐6 inhibits IGF‐II‐induced cell proliferation, differentiation, migration and survival. The binding of IGF‐II to the IGF‐IIR/CI‐MPR (IGF receptor type II/cation‐independent mannose 6‐phpsphate receptor) is also shown leading to IGF‐II internalization and degradation. The double arrows underpin the equilibrium between IGF‐II‐bound and IGF‐II‐unbound IGFBP‐6 IGF receptors. IGFBP‐6 binding to prohibitin‐2 (PBH2) mediates IGF‐independent inhibition of cancer cell migration induced by IGFBP‐6. Other IGF‐independent actions of IGFBP‐6 are inhibition of angiogenesis, inhibition of fibroblast proliferation and induction of apoptosis. Recent evidences support that IGFBP‐6 has also a regulatory role in the immune system by inducing chemotaxis of T cells, monocytes and neutrophils (PMN), as well as by increasing oxidative burst of neutrophils. All these actions are mediated by unknown receptors. The shown protein structures of IGFBP‐6, IGF‐I, IGF‐II and IGF receptors were taken and pictorially modified from the RCSB‐protein data bank (http://www.rcsb.org/). See text for further details

**Figure 3:** Intracellular actions of IGFBP‐6. IGFBP‐6 is shown to be imported into the nucleus, via an α‐importin‐mediated mechanism, where it binds to VDR (vitamin D receptor) interfering with formation of the transcription complex RXR (retinoid X receptor)/VDR. Further proven interactors of IGFBP‐6 are TRα1 (thyroid hormone receptor‐α1) and H2Br (histone cluster 1 H2br). Moreover, IGFBP‐6 can bind to the promoter of EGR‐1 (early growth response‐1). In the cytoplasm, IGFBP‐6 is shown to affect the nuclear import of Ku80 (Lupus Ku autoantigen protein p80) involved with Ku70 in NHEJR (non‐homologous end join repair). In addition, it hypothesized the interaction between IGFBP‐6 and the mitochondrial PHB1/2 (prohibitions 1 and 2) complex. See text for further details

As hyperthermia could induce an increased expression of IGFBP‐6 by at the level of dendritic cells (DCs), as well as their metabolic reprogramming, we are currently testing the ability of IGFBP‐6 to induce metabolic reprogramming in DCs. The implications of all these findings for cancer biology and pathogenesis of inflammatory disorders are further discussed below.

The article "From fever to immunity: A new role for IGFBP‐6?" was published in 2018. Journal: J Cell Mol Med.

## 4 THE IGF SYSTEM, IGFBP‐6 AND CANCER

The involvement of the IGF system in cancer is multifaceted. IGFs in general and IGF‐II in particular are involved in promoting tumour growth in situ in an autocrine or paracrine fashion once the tumour has been established. Many cancers overexpress *IGF2* 59 by mechanisms including loss of imprinting (LOI) and loss of heterozygosity (LOH).^60^, ^61^ Interestingly, other observations indicate that the IGF system might be important also for tumour cell death. IGF‐IIR/CI‐MPR acts as a receptor for intracellular lysosomal enzymes and, importantly, for granzyme B, a mediator of CTL‐induced apoptosis of target cells.^26^ These findings may implicate that tumours carrying non‐functional IGF‐IIR/CI‐MPR would have also an inherent resistance to CTLs, implying the development of novel strategies of immunotherapy of cancer.

As we have outlined above, the role of IGFBP‐6 in cancer is complex and stems from its primary role as a modulator of IGF‐II bioavailability and hence as a negative regulator of cancer cell growth. Indeed, it has been considered a tumour suppressor gene. On the other hand, IGFBP‐6 inhibits angiogenesis and induces apoptosis of cancer cells in an IGF‐independent manner.^25^ Moreover, IGFBP‐6 promotes cancer cell migration (see below).

## 5 CELL MIGRATION AND CHEMOTAXIS IN TUMOUR MICROENVIRONMENT

The tumour microenvironment (TME) plays a fundamental role in tumour cells’ acquirement of cancer hallmarks, thus being involved in cancer formation but also in its progressive and invasive phases.^62^, ^63^ Many cellular components are part of the TME, including fibroblasts, myofibroblasts, neuroendocrine cells, adipose cells, immune‐inflammatory cells, and the lymphatic and blood vascular network. Stemming from the historical definition that “cancer is a wound that does not heal”,^64^ it has been comprehended that indeed inflammation and immune response in the tumour microenvironment have many cancer promoting effects.^65^, ^66^ They are implicated in direct supply of mitogenic signals, modification of the ECM by proteases and thus uncaging bioactive mitogenic agents, cleavage of cell–cell and cell–ECM adhesion molecules, binding to tumour cells avoiding their apoptotic response, induce and foster angiogenesis, invasion and metastasis.

The article "From fever to immunity: A new role for IGFBP‐6?" was published in 2018. Journal: J Cell Mol Med.

A complex network of chemokines regulates chemotaxis of tumour cells in TME, and both cancer and inflammatory cells produce several cytokines and chemokines that attract and activate tumor‐infiltrating cells, including tumour‐associated macrophages (TAMs) and T cells.^67^ Several major events are affected by chemotaxis in the context of the TME: immune evasion, angiogenesis, invasion and dissemination. For example, CCL2 (MCP‐1) and CCL5 (RANTES) are major attractants of monocyte precursor cells in tumours and, when accumulated, these cells play an important part in tumour non‐responsiveness by suppressing antigen‐specific T cell responses.^68^

IGFBP‐6 is likely involved in the attraction of inflammatory and immune cells in this context.^25^ Previous studies have shown that in both normal and cancer cells, IGFBP‐6 impairs migration by inhibiting IGF‐II actions^40^, ^41^, ^42^ and by promoting EGR (early growth response protein)‐1 transcription in an IGF‐independent manner.^51^ On the other hand, IGFBP‐6 promotes rhabdomyosarcoma (RMS) cell migration by an IGF‐independent mechanism that involves MAPK pathway activation.^69^, ^70^ These results raised the possibility that a receptor or membrane protein may be involved. It was further demonstrated that prohibitin‐2 (PBH2) binds IGFBP‐6 on the cell surface of RMS cells.^58^ Although PBH2 was indispensable for IGFBP‐6‐induced cell migration, this action was not dependent on MAPK activation. Therefore, PBH2 is essential for IGFBP‐6‐induced RMS migration either by acting as a downstream effector of MAPKs or regulating migration independently of MAPK activation. Which cell type is producing IGFBP‐6 to attract tumour cells is not clear yet.

IGF‐II, wild‐type (wt) and mutated IGFBP‐6 were shown to determine alteration in the migration of ovarian cancer cells.^71^ IGFBP‐6 increased migration of SKOV3 ovarian cancer cells (transitional phenotype) in an IGF‐independent manner. However, IGFBP‐6 inhibited migration of HEY ovarian cancer cells (aggressive phenotype). As IGF‐II reversed the inhibitory effects of wt but not mutant IGFBP‐6 in HEY cells, these data suggest that IGFBP‐6 inhibited migration by both IGF‐dependent and IGF‐independent mechanisms. MAP kinases, and in particular the JNK and ERK pathways, were partially implicated in these effects on both cell lines, so that this involvement cannot explain the opposite direction of the migratory responses. It should be further investigated whether a differential molecular landscape, linked to a different phenotype, might be underlying the differential effects of IGFBP‐6 on migration of these cells. Overall, these results indicate that IGFBP‐6 effects on migration of tumour cells are based strongly on the tumorigenesis stage, although this should be corroborated by in vivo evaluation of tumour behaviour.

The article "From fever to immunity: A new role for IGFBP‐6?" was published in 2018. Journal: J Cell Mol Med.

## 6 IGFBP‐6 NEW ROLE IN THE INFLAMMATORY RESPONSE AND INFLAMMATORY DISORDERS

Inflammation and innate immunity are complex phenomenon that are apparently redundant but that may be evolutionarily driven to comply with encounters with diverse damaging and infectious agents.^72^ These defensive responses may be eventually subverted in cancer and autoimmune diseases by a wealth of mechanisms,^73^ including macrophage and neutrophil plasticity, and loss of immunological tolerance mediated by DCs.^74^

Neutrophils are the main cell type involved in the acute inflammatory response. Upon bacterial product release or cytokine production, these cells are primed in the circulation, are attracted into the inflamed tissue where they exert their main defence actions by phagocytosis, ROS production and release of the their granule content.^75^, ^76^ While neutrophil elastase (NE) and myeloperoxidase (MPO) are stored in primary granules, tertiary granules are enriched with metalloproteases (MMPs), in particular MMP‐9.^77^ At the mucosal level, this multi‐step process leads to migration across the endothelium, the extracellular matrix and the epithelium because of a chemoattractant gradient.^78^ We recently investigated whether IGFBP‐6 could have any effect on neutrophils’ functions as diverse ROS production, degranulation and chemotaxis.^23^ IGFBP‐6 induced a significant increase in ROS production in neutrophils obtained from healthy donors at all the concentrations tested as compared to untreated controls, with a peak obtained at 1 μg/mL. In relation to degranulation, IGFBP‐6 increased significantly MPO levels but did not modify MMP‐9 levels as compared to controls. Finally, IGFBP‐6 was tested as chemoattractant in a polarized model of airway epithelium in the physiologically relevant mode, that is, adding neutrophils to the basolateral side of the epithelium and IGFBP‐6 to the apical side.^79^ Under these experimental conditions, IGFBP‐6 attracted neutrophils maximally at the concentrations of 0.1 and 1 μg/mL. The addition of known agonists of neutrophils’ function, such as phorbol myristate acetate (PMA) or N‐formylmethionyl‐leucyl‐phenylalanine (fMLP), after IGFBP‐6 incubation did not exert any synergistic effect, indicating that IGFBP‐6 does not act as primer for neutrophils and suggesting that it might exert its action through the same signal transduction pathways elicited by either PMA or fMLP, including phospholipase C (PLC), phosphatidylinositol 3‐kinase (PI3K), and Src‐family kinases for fMLP,^80^, ^81^ and protein kinase C for PMA.^82^

The article "From fever to immunity: A new role for IGFBP‐6?" was published in 2018. Journal: J Cell Mol Med.

Recently, we have shown that IGFBP‐6 has chemoattractant properties towards monocytes and T cells but not B cells.^21^ Recombinant IGFBP‐6 increased monocyte migration in a dose‐dependent fashion to a maximum of 187 ± 31% of control (*P* < .05 as compared to cells migrating in the absence of IGFBP‐6). T cell chemotaxis was also significantly increased, showing a peak at 4 nmol/L (0.1 μg/mL; 180 ± 29% of control, *P* < .05), with a behaviour similar to SDF‐1. Concentrations of IGFBP‐6 lower than 4 nmol/L had no chemotactic activity for T cells. The specificity of the chemotactic effect was shown by the preincubation of IGFBP‐6 with an anti‐IGFBP‐6 antibody that abolished its chemotactic activity.

Rheumatoid arthritis (RA) is a chronic inflammatory disorder, where pannus development and cartilage and bone damage at the joint level recall tumour development and invasion. In a recent study,^22^ we have shown that IGFBP‐6 serum levels are higher in RA than in healthy controls and patients with osteoarthritis (OA). On the other hand, RA synovial fluid (SL) and synovial tissue (ST) presented lower and higher levels of IGFBP‐6 as compared to OA SL and ST, respectively. High levels of IGFBP‐6 in ST may be relevant for immune cell chemoattraction into the inflamed synovia; indeed, in vitro experiments confirmed that IGFBP‐6 acts as chemoattractant for RA immune cells, in particular T lymphocytes, and that this effect was partially inhibitable by dexamethasone. Intriguingly, infiltrating monocytes and fibroblasts expressed IGFBP‐6, likely pointing out to these cell types as the source for IGFBP‐6 in the context of inflamed synovia.

## 7 CONCLUSION

In summary, recent findings are consistent with the emerging notion that any immunological response to external stimuli needs to cope with a specific metabolic rewiring of the immunocompetent cells. The consequence of hyperthermic stress discussed here in MoDCs, mimicking physiological febrile temperatures in humans, unveiled that the sole physical input is sensed as an alert stimulus triggering a transition in dendritic cells from a quiescent state into a pre‐activated state. Such a transition occurs in a narrow temporal window and is accompanied by a significant change in the metabolic reprogramming which therefore is a very early event in the immune response functioning.

The article "From fever to immunity: A new role for IGFBP‐6?" was published in 2018. Journal: J Cell Mol Med.

Finally, IGFBP‐6 seems to play an important role in the control of cell‐specific immunologic adaptation following hyperthermia. In vivo experiments are warranted to fully explore the role of IGFBP‐6 in pathology and to discover how we might exploit its functions in diagnosis and therapy.

## CONFLICT OF INTEREST

The authors declare no conflict of interest.
